The article "MRI Findings of Pituitary Gland in Growth Hormone-Deficient Children and Their Correlation with Growth Hormone Peak during Growth Hormone Stimulation Tests" was published in 2022. Journal: Contrast Media Mol Imaging.

# MRI Findings of Pituitary Gland in Growth Hormone-Deficient Children and Their Correlation with Growth Hormone Peak during Growth Hormone Stimulation Tests

**DOI:** 10.1155/2022/3111585

**Published:** 2022-08-10

**Authors:** Jun Chen, Xiaofei Wang, Chengyong He, Siwen Wei

**Affiliations:** ^1^Department of Radiology, Xi'an Peoples Hospital (Xi'an Fourth Hospital), Xi'an 710004, Shanxi, China; ^2^Department of Radiology, Xi'an Children's Hospital, Xi'an 710003, Shanxi, China

## Abstract

This study aims to explore the magnetic resonance imaging (MRI) findings of the pituitary gland (PG) in children with growth hormone deficiency (GHD) and their correlation with the growth hormone (GH) peak during clinical GH stimulation tests. Sixty-one children with GHD diagnosed and treated between December 2018 and December 2021 were retrospectively analyzed in terms of clinical and pituitary morphological MRI data. MRI measurements of various diameters of the adenohypophysis (AH) were obtained to analyze the differences of the measured values in different genders and age groups, as well as their relationship with the GH peak in GH stimulation tests. Among the 61 children with GHD, the superior PG margin was protuberant in 2 cases, flat in 13 cases, and concave in 46 cases. The three age groups showed similar pituitary morphology and stalk (*P* > 0.05). On T1-weighted images, the proportion of isointensity was lower while the proportion of slightly-low signal intensity was higher in the anterior pituitary gland (APG) of children aged >10 compared with those aged 7–10. The comparison of AH linear parameters and GH peak values of male patients among different age groups showed that the anteroposterior (sagittal) diameter of AH and GH peak were the highest in the >10-year-old group and the lowest in the ≤6-year-old group, with those of the 7–10-year-old group in between (*P* < 0.05). In females, the anteroposterior (sagittal) diameter and GH peak were higher in the 7–10-year-old group and >10-year-old group compared with the ≤6-year-old group (*P* < 0.05). The MRI coronal and sagittal heights of PG in children with GHD were positively correlated with the GH peak value. In conclusion, in GHD patients, the coronal and sagittal heights as well as the coronal width of AH do not change with sex or age, but the coronal and sagittal heights of PG are positively correlated with the GH peak of GH stimulation tests, which has high application value in the diagnosis of children with GHD.

## 1. Introduction

Growth hormone deficiency (GHD) is a common growth and development disorder in clinical practice, which is triggered by a partial or complete deficiency of growth hormone (GH) synthesis and secretion in the anterior pituitary gland (APG) or by receptor defects and structural abnormalities [1]. With an ever-higher incidence worldwide, childhood GHD has become one of the major health issues affecting children in developing countries [2]. Relevant evidence shows an incidence of about 1/30,000 in terms of childhood GHD [3], which is higher than that of adult GHD, about 1.2/100,000 [4]. The health of children with GHD is more concerning, as children are more vulnerable [5, 6]. Growth failure, which is manifested in short stature and height below the third percentile of the growth curve of normal healthy children of the same age and sex, or two standard deviations below normal, is the main feature of GHD, which may affect the quality of life and psychosocial development of the affected children [7–9]. Clinically, it is believed that the earlier the patient is treated, the better the effect, so early diagnosis of GHD is of great significance to children.

The article "MRI Findings of Pituitary Gland in Growth Hormone-Deficient Children and Their Correlation with Growth Hormone Peak during Growth Hormone Stimulation Tests" was published in 2022. Journal: Contrast Media Mol Imaging.

The current diagnosis of GHD is primarily based on nutritional criteria and laboratory investigation, including testing for GH secretion by stimulating GH release [10]. As for nutritional criteria, “severe” short stature is defined as height < -3 standard deviation (SD) below the mean, height < -1.5 SD below the midparental height, and height < -2 SD below the mean, with either height velocity < -1 SD below the mean over the past year or height SD decreasing by more than 0.5 SD over the past year. Neonatal signs and symptoms of GHD include hypoglycemia, prolonged jaundice, microphallus, or craniofacial midline abnormalities [10]. The identification of central nervous system (CNS) tumors remains the primary purpose of neuroradiology in evaluating GHD children. Brain magnetic resonance imaging (MRI) plays a secondary role in identifying pituitary anatomical abnormalities that can aid clinicians in their diagnosis and prognosis [11]. With the advancement of medical imaging technology, MRI can be used to clearly display the morphology of the pituitary gland (PG), identifying hypoplastic anterior pituitary (HAP), ectopic posterior pituitary (EPP), pituitary stalk dysplasia, atrophy, etc., which has a wide range of applications in the diagnosis of pituitary abnormalities. The Growth Hormone Research Society (GRS) currently recommends that any child diagnosed with GHD should undergo an MRI examination of the brain, with particular attention to the hypothalamic-pituitary region [10]. However, previous studies have been inconclusive, showing a wide variation in the prevalence of MRI abnormalities among GHD patients, ranging from 25.9% to 100.0% [12–14]. There are also clinical reports showing some imaging changes in the PG of GHD children, including HAP, EPP, hypoplasia, interruption of pituitary stalk, etc. [11]. Because of this variability, patients with mild GH values are less likely to undergo brain MRI. Moreover, in clinical settings, some healthcare providers will only perform brain MRI examinations when patients have severe GHD or other risk factors like other pituitary hormone deficiencies, severe headaches, or vision problems.

The article "MRI Findings of Pituitary Gland in Growth Hormone-Deficient Children and Their Correlation with Growth Hormone Peak during Growth Hormone Stimulation Tests" was published in 2022. Journal: Contrast Media Mol Imaging.

Therefore, we measured PG size on MRI in GHD children in this study, observed the MRI manifestations of the pituitary morphology, and analyzed the correlation between PG measurements and the GH peak in GH stimulation tests, so as to provide a reference for the diagnosis and treatment of children with GHD.

## 2. Data and Methods

### 2.1. General Information

The clinical data and pituitary morphological MRI data of 61 children diagnosed with GHD (33 males and 28 females; 4–18 years old) presented to the Xi'an Peoples Hospital (Xi'an Fourth Hospital) from December 2018 to December 2021 due to short stature were retrospectively analyzed. Inclusion criteria were as follows: (1) in accordance with relevant diagnostic criteria for GHD [15]; (2) normal weight and body length at birth; (3) serum GH peak <10 *μ*g/L in more than two GH stimulation tests; (4) bone age 2 years younger than the chronological age; (5) short stature, with a height 2 standard deviations lower than normal children of the same sex and age; (6) no previous GH therapy; and (7) complete clinical data such as imaging data. Exclusion criteria were as follows: (1) slow growth and development due to other reasons; (2) moderate or severe infectious diseases; (3) hematopoietic or coagulation dysfunction; (4) organic diseases or severe malnutrition; and (5) incomplete clinical data such as imaging material. This Ethics Committee approved this study.

### 2.2. Inspection Methods

All the enrolled children underwent routine physical examinations after admission. In addition, 3 mL of venous blood was collected on an empty stomach for GH stimulation tests that were conducted over two days. On the first day of the test, all the children were given arginine hydrochloride intravenously. This was completed within 30 minutes, with a dosage of 0.5 g/kg (diluted into a 10% solution with normal saline) and a maximum dosage of 30 g. The next day, the children were given oral clonidine hydrochloride tablets (Changzhou Pharmaceutical Factory Co., Ltd., SFDA Approval No. H32021681, Specification: 75 *μ*g*∗*100 tablets) at a dosage of 5 *μ*g/kg, with a maximum of 250 *μ*g. Serum GH values of children in both groups were detected before, as well as 30 min, 60 min, and 90 min after administration, and the GH peak values were recorded.

The article "MRI Findings of Pituitary Gland in Growth Hormone-Deficient Children and Their Correlation with Growth Hormone Peak during Growth Hormone Stimulation Tests" was published in 2022. Journal: Contrast Media Mol Imaging.

All subjects were examined by pituitary MRI. A 1.5 T MRI scanner was used to scan the coronal, sagittal T1WI, and coronal T2WI sequences, with the parameters set as follows: T1WI : TR 400 ms, TE 20 ms; T2WI : TR 3000 ms, TE 90 ms; matrix: 288 × 192; slice thickness 2 mm; field of view (FOV): 18 cm × 18 cm, and; number of excitations: 2–3. Gd-DTPA contrast agent was used for enhancement, with a dose of 0.2 mL/kg and a concentration of 0.05 mmol/mL. After scanning, two highly qualified radiologists retrospectively reviewed the MRI images to observe the MRI features of the PG in GHD children, as well as superior pituitary morphology and pituitary signal characteristics.

### 2.3. Endpoints

1. The morphology of PG and pituitary stalk were observed. Pituitary morphology is divided into three types according to the median sagittal view, namely, concave, flat, and protuberant.
2. Linear parameters of the adenohypophysis (AH), including coronal height, coronal width, sagittal height, and sagittal anteroposterior diameter, were determined. On the midsagittal plane, the sagittal height (the height of the vertical-horizontal line at the midpoint of AH) and the sagittal anteroposterior diameter (the horizontal linear distance between the anterior and posterior edges of AH) of AH were measured. On the coronal plane, the coronal height (vertical height and horizontal distance from the pituitary midpoint) and coronal width (horizontal line distance between the left and right edges of the PG) of AH were tested. The values of the linear parameters measured were averaged after two measurements.

### 2.4. Statistical Analysis

Data analysis was performed by SPSS 20.0, and the significance level in this study is *P* < 0.05. Inter-group differences of quantitative data denoted by mean ± mean were identified using an independent sample *t*-test, while multigroup differences were determined via one-way ANOVA, followed by a Bonferroni post-hoc test. The *χ*^2^ test was adopted for categorical data represented by *n* (%). Pearson's Linear Correlation was used for correlation analysis between variables.

## 3. Results

### 3.1. MRI Manifestations and Signal Characteristics of PG

The observation showed no statistical differences in pituitary morphology and stalk among the three age groups (*P* < 0.05). On T1-weighted images, the proportion of isointensity was lower while the proportion of slightly-low signal intensity was higher in the APG of children aged >10 compared with those aged 7–10, with statistical significance (*P* < 0.05, Table 1). Adenohypophysial atrophy was observed on sagittal T1WI and coronal enhanced T1WI in one child. An absent pituitary stalk is shown in Figure 1.

The article "MRI Findings of Pituitary Gland in Growth Hormone-Deficient Children and Their Correlation with Growth Hormone Peak during Growth Hormone Stimulation Tests" was published in 2022. Journal: Contrast Media Mol Imaging.

### 3.2. MRI Measurements of PG

No statistical differences were found in various PG linear parameters between male and female patients of the same age group (*P* > 0.05). The comparison (Table 2) of AH diameters of male patients among different age groups showed that the PG anteroposterior (sagittal) diameter was the highest in the >10-year-old group and the lowest in the ≤6-year-old group, compared with those of the 7–10-year-old group in between (*P* < 0.05). In females, the anteroposterior (sagittal) diameter was higher in the 7–10 and >10-year-old groups compared with the ≤6-year-old group (*P* < 0.05).

### 3.3. GH Peak in GH Stimulation Tests in Children

There was no significant difference in the peak GH value in GH stimulation tests between different sexes of the same age group (*P* > 0.05). The comparison of the GH peak in male patients among different age groups showed that the peak GH value was the highest in the >10-year-old group, followed in descending order by the 7–10-year-old group and the ≤6-year-old group (*P* < 0.05); and in female patients of different age groups, the peak GH value was significantly higher in the 7–10-year-old group and > the 10-year-old group compared with the ≤6-year-old group (*P* < 0.05).  Table 3.

### 3.4. Correlation Analysis between MRI Measurements of PG and GH Peak in Stimulation Tests

MRI findings revealed a positive association between sagittal and coronal heights of PG and GH peak in stimulation tests in children with GHD (*r* = 0.2541, *P*=0.0482; *r* = 0.3428, *P*=0.0068); while no significant correlation was determined between coronal width, sagittal anteroposterior diameter, and GH peak (*P* > 0.05), as shown in Figure 2.

## 4. Discussion

Clinically, GHD can be divided into primary and secondary GHD, of which the former is mostly associated with heredity, idiopathic hypothalamic dysfunction, and dysplasia [16, 17], while the latter is mainly related to tumors, radiation injury, and head trauma [18, 19]. Primary GHD occurs most frequently in preadolescent children, often presenting with growth retardation and loss of appetite. The treatment difficulty of this disease is directly proportional to the amount of time, and without timely intervention, it will eventually seriously affect the lives of children. Therefore, early diagnosis and treatment are of great significance to children's physical and mental development.

With the continuous development of medical technology and the deepening of neuroimaging analysis methods in recent years, multimodal MRI technology makes it possible to conduct in-depth research on brain structure and function to a large extent and achieve rapid, convenient, and noninvasive results [20, 21]. It can help us better understand the influence mechanism of the disease on the human brain, so as to analyze the institutional basis of cognitive behavior from different perspectives and realize a comprehensive understanding of the relationship between hormones and brain structure from a dimensional perspective by combining our laboratory data collection of hormone levels. Our research results showed no significant difference in pituitary morphology and stalk among the three age groups. However, children aged over 10 showed a lower proportion of T1 isointensity and a higher proportion of slightly lower T1 signal intensity than those aged 7–10. Pituitary height is known to effectively reflect APG development. Under normal circumstances, the volume and shape of PG will gradually change with age, among which flat PG is the most commonly seen [22, 23]. The area of PG grows accordingly as age increases, which makes the upper edge of PG bulge outwards gradually. The results of this study showed that the superior pituitary border of GHD children was mainly concave while rarely protuberant, with some cases presenting a flat superior PG border. Generally, the MRI signals of the APG are similar to those of the brain stem. However, due to the decreased function of APG to synthesize hormones in GHD children and reduced pituitary volume compared with that of healthy people, a volume effect is produced between the APG and the low signal of the surrounding cerebrospinal fluid. With age, HAP in GHD children is getting worse, resulting in a decreased T1 signal in APG [24], similar to the study of Xu et al. [25]. In addition, GHD patients are often accompanied by insufficient gonadal hormone secretion in addition to GH secretion insufficiency, which leads to abnormal development of PG due to a lack of adequate doses of sex hormones during growth and development.

The article "MRI Findings of Pituitary Gland in Growth Hormone-Deficient Children and Their Correlation with Growth Hormone Peak during Growth Hormone Stimulation Tests" was published in 2022. Journal: Contrast Media Mol Imaging.

In recent years, a large amount of research data has confirmed that the height of PG in children, which can effectively reflect the development of APG, is positively correlated with their age [22, 26]. Generally speaking, as the pituitary volume increases with age, the adenohypophysial diameter gradually increases, among which the height changes most obviously. In this study, the sagittal anterior-posterior diameter and GH peak in GH stimulation tests were compared among children of different sexes and age groups. Among males, the sagittal anterior-posterior diameter and GH peak were the highest in children aged >10, followed in descending order by 7–10 and ≤6 age groups. And in female patients, the sagittal anteroposterior diameter and GH peak were higher in the 7–10-year-old group and > the 10-year-old group compared with the ≤6-year-old group. There is a positive linear relationship between normal pituitary size and age, with gender differences. During puberty, pituitary diameters change significantly, especially with the increase in height. However, the poor development of APG in children with GHD leads to the decline of adenohypophysial function, which in turn reduces the level of GH in the body, resulting in a relatively small pituitary volume. This result is basically consistent with the findings of Gustavo et al. [27].

Finally, by comparing GH stimulation test results among different groups of children, we found that the coronal and sagittal heights of pituitary MRI in children with GHD were positively correlated with the GH peak in GH stimulation tests. GH, as an important peptide hormone synthesized and secreted by the APG, enters the blood and binds with the GH binding protein (GHBP) of the body to be transported to various target organs [28]. GH has various physiological functions, mainly using the mediation of insulin-like growth factors to play its role in promoting growth. As GH in human blood shows a pulsatile secretion pattern [29], it is necessary to conduct a GH stimulation test when detecting GH. This study compared the peak GH in GH stimulation tests of male patients of different ages and found that the peak GH was the highest in the >10-year-old group and the lowest in the 7–10-year-old group, with that in the ≤6-year-old group in between. In female patients, the GH peak was statistically higher in the 7–10-year-old group and > the 10-year-old group compared with the ≤6-year-old group. Thus, the stimulating peak of GH is different in children of different ages. In addition, the coronal and sagittal heights of pituitary MRI in children with GHD were found to be positively correlated with the GH peak. In childhood, the mature hypothalamus-pituitary-target organ feedback system allows for gradual proliferation of AH cells, causing enhanced secretion of multiple hormones and increased pituitary volume, with a positive connection between the two [30].

To sum up, MRI has a favorable diagnostic effect in GHD patients and can clearly display the pituitary morphological characteristics. The coronal height, sagittal height, and coronal width of PG in GHD patients do not change with sex or age, but the coronal and sagittal heights of PG are positively correlated with the GH peak in GH stimulation tests. These results provide an objective reference for the clinical treatment of GHD.

## Figures and Tables

**Figure 1:** MRI image of the same child. (a) Sagittal T1WI image and (b) coronal T1WI image.

The article "MRI Findings of Pituitary Gland in Growth Hormone-Deficient Children and Their Correlation with Growth Hormone Peak during Growth Hormone Stimulation Tests" was published in 2022. Journal: Contrast Media Mol Imaging.

**Figure 2:** Correlation analysis between pituitary MRI measurements and GH peak in stimulation tests. (a) Correlation between sagittal height and GH peak in stimulation tests; (b) correlation between crown height and GH peak in stimulation tests; (c) correlation between crown width and GH peak in stimulation tests; and (d) correlation between sagittal anteroposterior diameter and GH peak in stimulation tests.

**Table 1:** Pituitary manifestations of all children.

Age (years)	Pituitary morphology *n* (%)			Signal intensity *n* (%)		Pituitary stalk *n* (%)	
	Concave	Flatt	Protuberant	T1 isosignals in anterior pituitary	T1 slightly-low signal intensity	Hypoplasticc	Absent
≤6 (*n* = 15)	11	4	0	11	4	2	0
7–10 (*n* = 33)	26	6	1	26	7	6	10
>10 (*n* = 13)	9	3	1	4^*∗*^^#^	9^*∗*^^#^	6	4

Note: ^*∗*^*P* < 0.05 vs. ≤6-year-old group; ^#^*P* < 0.05 vs. 7–10-year-old group.

**Table 2:** Statistics of adenohypophyseal linear parameter in different gender and age groups.

	Male (*n* = 33)			Female (*n* = 28)		
	≤6 (*n* = 9)	7–10 (*n* = 15)	>10 (*n* = 9)	≤6 (*n* = 6)	7–10 (*n* = 18)	>10 (*n* = 4)
Coronal height (mm)	2.77 ± 1.16	3.08 ± 1.55	3.90 ± 1.60	2.97 ± 1.05	3.03 ± 1.48	4.26 ± 1.62
Coronal width (mm)	8.81 ± 1.02	9.47 ± 1.97	10.14 ± 1.52	8.63 ± 0.96	9.56 ± 1.97	10.07 ± 1.71
Sagittal height (mm)	2.68 ± 0.63	3.55 ± 1.20	4.24 ± 1.26	2.91 ± 0.47	3.56 ± 1.23	4.50 ± 1.44
Sagittal anteroposterior diameter (mm)	5.71 ± 0.78	6.25 ± 1.11^*∗*^	7.02 ± 1.17^*∗*^^#^	5.42 ± 0.77	6.11 ± 1.11^*∗*^	6.93 ± 1.04^*∗*^

Note. Within the group, ^*∗*^*P* < 0.05 vs. ≤ 6-year-old group; ^#^*P* < 0.05 vs. 7–10-year-old group.

**Table 3:** Peak growth hormone value in growth hormone stimulation tests.

	Male (*n* = 33)			Female (*n* = 28)		
	≤6 (*n* = 9)	7–10 (*n* = 15)	>10 (*n* = 9)	≤6 (*n* = 6)	7–10 (*n* = 18)	>10 (*n* = 4)
Peak GH value after stimulation (*μ*g/L)	1.06 ± 0.88	2.19 ± 0.91^*∗*^	3.26 ± 0.73^*∗*^^#^	1.18 ± 0.50	2.35 ± 1.04^*∗*^	3.31 ± 1.00^*∗*^

Note. ^*∗*^*P* < 0.05 vs. ≤6-year-old group; ^#^*P* < 0.05 vs. 7–10-year-old group.

## Data Availability

The labeled dataset used to support the findings of this study are available from the corresponding author upon request.
